# LINC01089 functions as a ceRNA for miR-152-3p to inhibit non‐small lung cancer progression through regulating PTEN

This article has been retracted.

**DOI:** 10.1186/s12935-021-01846-7

**Published:** 2021-03-02

**Authors:** Huixian Zhang, Hao Zhang, Xingya Li, Siyuan Huang, Qianqian Guo, Di Geng

**Affiliations:** 1 Department of Oncology, The First Affiliated Hospital of Zhengzhou University, Νo.1 Jianshe East Road, Zhengzhou, 450052 Henan China; 2 Department of Radiology, Changhai Hospital Affiliated to The Second Military Medical University, No.168 Changhai Road, Shanghai, 200433 China

**Keywords:** LINC01089, NSCLC, miR-152-3p, PTEN

## Abstract

**Background:**

Long non-coding RNAs (lncRNAs) have been reported to exert crucial functions in regulating the progression of human cancers. However, the function and mechanism of long intergenic non-protein coding RNA 01089 (LINC01089) in non-small cell lung cancer (NSCLC) have not been revealed.

**Methods:**

The expression level of LINC01089, microRNA (miRNA, miR)-152-3p and phosphatase and tensin homolog deleted onc hromosome ten (PTEN) mRNA was detected by quantitative real-time PCR (qRT-PCR). After gain-of-function and loss-of-function models were established with NSCLC cell lines, the proliferation, migration and invasion of NSCLC cells were detected by cell counting kit-8 (CCK-8) assay, scratch healing assay, Transwell assay, respectively. Dual luciferase reporter assay was employed to validate the binding relationship between miR-152-3p and LINC01089 or the 3’UTR of PTEN. Western blot was used to detect PTEN expression in NSCLC cells after LINC01089 and miR-152-3p were selectively modulated.

**Results:**

LINC01089 was down-regulated in NSCLC tissues and cells. Functional experiments showed that knockdown of LINC01089 could promote the proliferation, migration and invasion of NSCLC cells, while over-expression of LINC01089 had the opposite effects. miR-152-3p was identified as a functional target for LIN01089, and miR-152-3p could reverse the function of LINC01089. Additionally, LINC01089 could up-regulate the expression level of PTEN via repressing miR-152-3p.

**Conclusions:**

Down-regulation of LINC01089 promoted the progression of NSCLC through regulating miR-152-3p/PTEN axis.

## Introduction

Lung cancer is a tumor with the highest morbidity and mortality worldwide [1–3]. Non-small cell lung cancer (NSCLC) is the principal type of lung cancer, accounting for about 80 % of all lung cancer cases [4]. In recent years, surgery, radiotherapy, chemotherapy and targeted therapy have made a great leap forward, but the overall survival time of NSCLC patients, especially those with distant metastasis and recurrence, was far from satisfactory [5]. The detailed mechanism of NSCLC progression still requires further investigation.

Long non-coding RNA (lncRNA) is named for its transcriptional length over 200 nucleotides and lacking protein coding ability. LncRNA is involved in multiple biological activities, like epigenetic regulation, cell cycle regulation and cell differentiation regulation [6–8]. It is revealed that lncRNA is abnormally expressed in a variety of tumors, and dysregulated lncRNAs are involved in cancer progression via a variety of mechanisms, including mediating chromatin remodeling and histone modification, binding with transcription factors and regulating their recruitment, and functioning as a precursor molecule of small RNA [9–12]. A recent study reports that LINC01089 is down-regulated in breast cancer, and it inhibits the invasion of breast cancer cells and its low expression is correlated with the poor prognosis of patients [13]. However the expression pattern, function and mechanism of LINC01089 in NSCLC awaits more investigation.

MicroRNA (miRNA) is a class of endogenous single-stranded non-coding RNA with approximately 19–25 nucleotides in length. MiRNAs can identify the specific target mRNAs and negatively modulate their expression at a post-transcriptional level via promoting degradation of them or inhibiting translational processes [14, 15]. miR-152-3p is cleaved from the precursor RNA transcribed from human chromosome 7q21.32, and the expression of miR-152-3p was down-regulated in prostate cancer and glioma, and its low expression was related to the low survival rate of patients [16, 17]. However, its function in NSCLC and its upstream and downstream mechanisms are still unclear.

Phosphatase and tensin homolog (PTEN) is one of the most famous tumor suppressors in cancer biology. Its deletion, down-regulation or mutation were observed in multiple human cancers [18, 19]. Additionally, PTEN is down-regulated in NSCLC tissues and can inhibit the progression of NSCLC via negatively regulating the PI3K-AKT-mTOR pathway [20]. In the present study, we demonstrated that LINC01089 is down-regulated in NSCLC tissues and cells. It was confirmed by gain-of-function and loss-of-function experiments that LINC01089 could impede the proliferation and metastasis of NSCLC cells. We also demonstrated that the defect of LINC01089 contributed to the down-regulation of PTEN in NSCLC, which is mediated by its regulation on miR-152-3p.

## Materials and methods

### Clinical samples

50 cases of NSCLC tissues and adjacent tissues were collected. None of the patients enrolled received anti-tumor therapy before surgery. All tissues were excised during surgery and immediately stored in liquid nitrogen at -196°C for subsequent experiments. This study was approved by the Ethics Committee of the First Affiliated Hospital of Zhengzhou University, and all the patients involved signed the informed consent.

### Cell culture

The China Center for Type Culture Collection (CCTCC, Chinese Academy of Sciences, Shanghai, China) was the provider of the cell lines used in this study. BEAS-2B cell, HCC827 cell, NCI-H460 cell, A549 cell, H1299 cell and HEK293T cell were cultured in Dulbecco’s Modified Eagle Medium (DMEM) (Thermo Fisher Scientific, Waltham, MA, USA) containing 10 % fetal bovine serum (FBS) (Thermo Fisher Scientific, Waltham, MA, USA) and 1 % penicillin/streptomycin (Invitrogen, Carlsbad, CA, USA). Cells were cultured in 5 % CO_2_ at 37 ℃ in a humidified incubator.

### Cell transfection

GenePharma Co.,Ltd. (Shanghai, China) was the provider of pcDNA empty vector (Vector), pcDNA-LINC01089 (LINC01089), shRNA normal control (sh-NC),shRNAs against LINC01089 (sh-LINC01089#1 and sh-LINC01089#2), miRNA control (NC-mim), miR-152-3p mimics, miR-152-3p inhibitors and inhibitors control (NC-in). HCC827 and H1299 cells were inoculated into a 24-well plate at a density of 3 × 10^5^ cells / well. Cells were cultured at 37 ℃ and 5 % CO_2_ for 24 h before transfection. In compliance with the supplier’s instructions, HCC827 and H1299 cells were transfected with Lipofectamine ®2000 (Invitrogen, Carlsbad, CA, USA). The transfection efficiency was determined by quantitative real-time polymerase chain reaction (qRT-PCR) 48 h after the transfection. The shRNA with better knockdown effect (sh-LINC01089#2) was selected for the following experiments.

### qRT-PCR

Total RNA was extracted from tissues and cells with TRIzol reagent (Thermo Fisher Scientific, Waltham, MA, USA). Reverse transcription was carried out using MMLV reverse transcriptase (Thermo Fisher Scientific, Waltham, MA, USA) to generate cDNA. On the ABI7500 real-time PCR system (Thermo Fisher Scientific, Waltham, MA, USA), qRT-PCR was operated using SYBR premix EX TAQ II (TaKaRa, Dalian,China) in compliance with the manufacturer’s instructions. GAPDH was used as the reference gene of LINC01089 and PTEN, and U6 was used as the reference gene of miR-152-3p. The relative gene expressions were calculated by 2^−ΔΔCt^ formula. Primers were designed using Primer 6.0 software. The specific primer sequences are: LINC01089 upstream primer: 5’-GCAGTAAACAGTCCTCAGCGAAG-3’, downstream primer: 5’-CGGTGCCATGGAGTCTAGAAGAT-3’;

miR-152-3p upstream primer: 5’-AGGGTCAGTGCATGACAGA-3’, downstream primer: 5’-TACCAACCAACCCACTCACT-3’;

PTEN upstream primer: 5’-AATTCCCAGTCAGAGGCGCTATGT-3’, downstream primer: 5’-GATTGCAAGTTCCGCCACTGAACA-3’;

U6 upstream primer: 5’-CGGGTGCTCGCTTCGCAGC-3’, downstream primer: 5’-CCA GTGCAGGGTCCGAGGT-3’;

GAPDH upstream primer: 5’-TATGATGATATCAAGAGGGTAGT-3’, downstream primer: 5’-TGTATCCAAACTCATTGTCATAC-3 ‘.

### CCK-8 assay

2 × 10^3^ cells in each group were inoculated into each well of a 96-well plate. After the cells were cultured for 24 h, 10 µL of CCK-8 solution (Dojindo, Kumamoto, Japan) was dripped into each well. The plate was then placed in the incubator for another 4 h, and then the absorbance value of the cells at 450 nm was measured by a microplate reader. Similarly, the changes in cell viability of the cells on the 2nd, 3rd, and 4th day were determined. Ultimately, the proliferation curve was plotted.

### Wound healing assay

Cells in the logarithmic growth phase were cultured in a 6-well plate at the density of 1 × 10^6^ cells / ml. When the cells reached 80% to 90% confluency, a sterile pipette was used to make a perpendicular scratch on the cells. Then the culture plate was washed three times with PBS, and the floating cells were removed, and then DMEM containing 2.5 % FBS was added, and the scratch was photographed under a microscope. After that, the cells were cultured in an incubator with 5 % CO_2_ at 37 ℃ for 24 h, and then the scratch was photographed again under the microscope. The migration ability of the cells was represented by the change of scratch width.

### Transwell assay

Transwell assay was used to detect cell invasion. The membrane of Transwell chamber (Corning, NY, USA) was coated with Matrigel. 2 × 10^4^ cells suspended in 200 µL of serum-free medium were added to the upper compartment of Transwell chamber, and 600 µL of medium containing 20 % FBS was loaded into the lower compartment. After cultured for 12 h, cells in the upper surface of the membrane were removed, and cells on the lower surface of the membrane was fixed in 4 % paraformaldehyde, stained with 0.1 % crystal violet, photographed and counted after drying. The cells were counted by naked eyes, assisted by Cell Counter (ImageJ, Rawak Software Inc., Germany). All counting was performed by researchers who were blinded to the groups.

### Western blot

The cells were collected and washed 3 times with cold PBS, and RIPA lysis buffer (Sigma-Aldrich, Shanghai, China) was added to extract the total protein. 5 µg of total protein in each group was applied to 12 % SDS-PAGE at 100 V for 2 h. Then the protein was electrotransferred to the PVDF membrane (Millipore, Bedford, MA, USA). The membrane was blocked with 5 % skim milk for 1 h at room temperature, washed 3 times for 10 min each time with TBST. Then the membrane was incubated with the primary antibodies anti-PTEN antibody [Y184] (ab32199, 1: 1000, abcam, Shanghai, China) and anti-GAPDH antibody (ab181602, 1: 2000, abcam, Shanghai, China) at 4 ℃ overnight. Next, the membrane was washed with TBST and was incubated with horseradish peroxidase (HRP)-labeled secondary antibody for 1 h at room temperature. Then the membrane was washed 3 times again with TBST for 10 min each time. Eventually, the bands were developed using ECL reagent (Millipore, Bedford, MA, USA).

### Dual luciferase reporter assay

The binding relationship between miR-152-3p and LINC01089 or the 3’-UTR of PTEN was confirmed by dual luciferase reporter method. Wild type (WT) LINC01089 sequence or the WT PTEN 3’-UTR sequence containing the predicted miR-152-3p binding site was amplified and inserted into the pmirGLO dual-luciferase miRNA target expression vector (Promega, Madison, WI, USA). The putative binding site of miR-152-3p in LINC01089 or PTEN 3’-UTR sequence was mutated using GeneArtTM Site-Directed Mutagenesis PLUS System (Thermo Fisher Scientific, Waltham, MA, USA). The mutant (MUT) LINC01089 or PTEN 3’-UTR sequence was inserted into the pmirGLO vector to construct the reporter vector pmirGLO-LINC01089-MUT or pmirGLO-PTEN-MUT. The corresponding reporter vector and miR-152-3p mimics or mimics-NC were co-transfected into HEK293T cells. After 48 h, the luciferase activity of the cells was measured using the Dual Luciferase Reporter Assay System (Promega, Madison, WI, USA) according to the manufacturer’s instruction.

### Statistical analysis

All data were analyzed using SPSS 22.0 software (SPSS Inc., Chicago, IL, USA). The results were expressed as mean ± standard deviation. Comparisons between the two groups were performed using an independent sample *t*-test. The association between pathological parameters and LINC01089 expression was tested by χ ^2^ test. *P* < 0.05 signified statistical significance.

## Results

### LINC01089 was lowly expressed in NSCLC tissues and it was correlated with poor prognosis

To delve into the expression characteristics of LINC01089 in NSCLC tissues and cells, we first demonstrated through the GEPIA database () that LINC01089 expression was dramatically down-regulated in both lung squamous cell carcinoma (LUSC) tissues and lung adenocarcinoma (LUAD) tissues compared with normal lung tissues (Fig. 1a, b). Moreover, we examined the expressions of LINC01089 in NSCLC tissues and cell lines by qRT-PCR. Being consistent with our expectations, qRT-PCR results displayed that LINC01089 expression was remarkably down-regulated in NSCLC tissues and cells (Fig. 1 c, d). Then we divided the NSCLC tissues into the LINC01089 high expression and low expression groups according to the median value, and analyzed whether LINC01089 can function as a prognostic marker. The results manifested that low expression of LINC01089 was correlated with increased tumor size, lymph node metastasis, and high TNM stage of the patients (Table 1). Additionally, GEPIA database indicated that underexpression of LINC01089 was associated with low survival rate in patients with NSCLC (Fig. 1e). These data suggested that LINC01089 was a tumor suppressor of NSCLC.

**Fig. 1:** Expressions of LINC01089 in NSCLC tissues and cells. **a**, **b**: The expression of LINC01089 in NSCLC tissues were analyzed using GEPIA database. Red column represented number of tumor samples, gray column represented number of normal samples. **c**: The expression of LINC01089 in NSCLC tissues was detected by qRT-PCR. ***P < 0.001. **d**: The expression levels of LINC01089 in normal lung epithelial cell line BEAS-2B and NSCLC cell lines were detected by qRT-PCR. *P < 0.05, **P < 0.01, ***P < 0.001. **e**: The association between LINC01089 expression and survival rate of NSCLC patients was analyzed by GEPIA database

**Table 1:** Correlation between LINC01089 expression and clinical features (n = 50)

Parameters	Group	n	LINC01089 expression		*P* value
			Low = 25	High = 25	
Gender	Male	23	9	14	0.157
	Female	27	16	11	
Age(years)	≦ 65	16	10	6	0.225
	> 65	34	15	19	
Tumor size	≦ 3 cm	23	16	7	0.011*
	> 3 cm	27	9	18	
Grade	Low	23	13	10	0.395
	High	27	12	15	
LNM	positive	31	12	19	0.041*
	negtive	19	13	6	
TNM stage	I	10	7	5	0.004**
	II	18	4	10	
	III	22	14	10	

*LNM* lymph node metastasis. * presents *P* < 0.05; ** presents *P* < 0.01

### LINC01089 inhibited NSCLC progression *in vitro*

Next, we established LINC01089 high and low expression cell models with NSCLC cell lines H1299 and HCC827, respectively. qRT-PCR was used to detect the transfection efficiency, and it indicated that the cell models were successfully constructed (Fig. 2a, b). We found through CCK-8 assay that high expression of LINC01089 markedly impeded the proliferation of H1299 cells, while knock down of LINC01089 promoted the proliferation of HCC827 cells (Fig. 2c, d). Then, cell migration and invasion assays were performed. We found that overexpression of LINC01089 blocked migration and invasion of H1299 cells, while knock down of LINC01089 had the opposite effects on HCC827 cells (Fig. 2e, f). These results manifested that LINC01089 can block the proliferation, migration and invasion of NSCLC cells as an tumor-suppressive lncRNA.

**Fig. 2:** Function of LINC01089 on proliferation, migration and invasion of NSCLC cells. **a**, **b**: qRT-PCR was used to detect the expression of LINC01089 after overexpression and knockdown of LINC01089 in NSCLC cell lines. ***P < 0.001. **c**, **d**: The proliferation of NSCLC cells after overexpression and knockdown of LINC01089 was detected by CCK-8 assay. *P < 0.05, **P < 0.01. **e**: The migration of NSCLC cells after overexpression and knockdown of LINC01089 was detected by scratch healing assay. *P < 0.05, **P < 0.01. **f**: Transwell assay was used to detect the invasive ability of NSCLC cells after LINC01089 was overexpressed or knocked down, *P < 0.05, **P < 0.01

### LINC01089 directly targeted miR-152-3p

Previous studies have shown that LINC01089 was mainly located in the cytoplasm of NSCLC cells [21], suggesting that it may function as a molecular sponge. To delve into the mechanism of LINC01089 in regulating the biological behaviors of NSCLC cells, we used bioinformatics analysis tool StarBase V2.0 () to screen the potential downstream targets for LINC01089. As shown (Fig. 3a), LINC01089 contained a conserved binding site for miR-152-3p. Pearson’s correlation analysis depicted that the expression of LINC01089 was negatively related with the expression of miR-152-3p in NSCLC tissues (Fig. 3b). To further validate the binding relationship between the two, we performed dual luciferase reporter assay. The assay demonstrated that the miR-152-3p mimics could decrease the luciferase activity of luciferase reporter containing LINC01089 WT, but exerted no significant effect on the luciferase activity of LINC01089 MUT reporter (Fig. 3c). Additionally, qRT-PCR indicated that overexpression of LINC01089 could down-regulate the expression level of miR-152-3p in NSCLC cells, while knockdown of LINC01089 had the opposite effect (Fig. 3d). Next, we examined the levels of miR-152-3p in NSCLC tissues and cells, and the results depicted that compared with para-cancerous tissues and lung epithelial cell line, the expression of miR-152-3p was remarkably up-regulated in NSCLC tissues and cell lines (Fig. 3e, f).

**Fig. 3:** There is a targeting relationship between LINC01089 and miR-152-3p. **a** It was found that LINC01089 contained a potential binding site for miR-152-3p, which was predicted by StarBase database. **b** Pearson’s correlation analysis was used to analyze the relationship between LINC01089 and miR-152-3p in NSCLC tissues. **c** The targeting relationship between LINC01089 and miR-152-3p was validated by dual luciferase reporter assay. NS *P* > 0.05, ***P < 0.001. **d** The expression of miR-152-3p in NSCLC cells after overexpression and knockdown of LINC01089 was detected by qRT-PCR. **P < 0.01, ***P < 0.001. **e** qRT-PCR was used to detect the expression of miR-152-3p in adjacent tissues and NSCLC tissues. ***P < 0.001, **f** The expression levels of miR-152-3p in normal lung epithelial cell BEAS-2B and NSCLC cell lines were detected by qRT-PCR. *P < 0.05, **P < 0.01

### MiR-152-3p promoted NSCLC progression in vitro

As mentioned above, we had proved that miR-152-3p was up-regulated in NSCLC. Then, to investigate the influence of miR-152-3p on the proliferation, migration and invasion of NSCLC cells, we established miR-152-3p over-expression and inhibition cell models with NSCLC cell lines HCC827 and H1299, respectively, and qRT-PCR was used to detect the transfection efficiency (Fig. 4a, b). We found through CCK-8 assay that over-expression of miR-152-3p significantly promoted the proliferation of HCC827 cells, while inhibition of miR-152-3p reduced the viability of H1299 cells (Fig. 4c, d). Then, wound healing assay and Transwell invasion assays were performed. It was demonstrated that over-expression of miR-152-3p promoted migration and invasion of NSCLC cells, while inhibition of miR-152-3p had the opposite effects (Fig. 4e, f). These results implied that miR-152-3p could promote the proliferation, migration and invasion of NSCLC cells as a cancer-promoting miRNA.

**Fig. 4:** The functions of miR-22-3p on proliferation, migration and invasion of NSCLC cells. **a**, **b** The expression of miR-152-3p was detected by qRT-PCR after transfection of miR-152-3p mimics and inhibitors. **P < 0.01, ***P < 0.001. **c**, **d** CCK-8 assay was used to detect the proliferation of NSCLC cells transfected with miR-152-3p mimics and inhibitors. *P < 0.05, **P < 0.01. **e** The migration ability of NSCLC cells transfected with miR-152-3p mimics and inhibitors was detected by wound healing assay. *P < 0.05. **f** Transwell assay was used to detect the invasive ability of NSCLC cells transfected with miR-152-3p mimics and inhibitors. *P < 0.05, **P < 0.01

### PTEN was a functional target of miR-152-3p

PTEN is down-regulated in NSCLC tissues, and it can function as a tumor suppressor and impede the proliferation and metastasis of NSCLC cells [20]. Interestingly, we searched five databases (microT, miRanda, miRmap, TargetScan, StarBase) for the potential target of miR-152-3p, and noticed that all of the five tools predicted that miR-152-3p could probably bind with the 3’UTR of PTEN mRNA(Fig. 5a). Pearson’s correlation analysis depicted that the expression of miR-152-3p in NSCLC tissues was negatively correlated with the expression of PTEN mRNA (Fig. 5b). To confirm the binding relationship between miR-152-3p and the 3’UTR of PTEN mRNA, dual luciferase reporter assay was employed. The results confirmed that the miR-152-3p mimics could reduce the luciferase activity of the luciferase reporter containing PTEN-WT, but had no significant effect on the luciferase activity of the PTEN-MUT reporter (Fig. 5c). In addition, Western blot manifested that compared with the control group, the expression of PTEN in NSCLC cells was markedly down-regulated after transfection of miR-152-3p mimics, and it was significantly increased after transfection of miR-152-3p inhibitors (Fig. 5d). After overexpression of LINC01089, the expression of PTEN in NSCLC cells was remarkably up-regulated (Fig. 5e); on the other hand, after knocking down LINC01089, the expression of PTEN was dramatically down-regulated (Fig. 5e). These results indicated that PTEN functioned as a target of miR-152-3p and it was positively modulated by LINC01089 in NSCLC.

**Fig. 5:** PTEN was a target gene of miR-152-3p. **a** The potential binding site between miR-152-3p and PTEN 3’UTR predicted by bioinformatics analysis. **b** Pearson’s correlation analysis of PTEN expression and miR-152-3p expression in NSCLC tissues. **c** The targeting relationship between PTEN and miR-152-3p was detected by dual luciferase reporter assay, NS *P* > 0.05, ***P < 0.001. **d** Western blot was used to detect the expression of PTEN in NSCLC cell lines after transfection of miR-152-3p mimics and inhibitors. **e** After overexpression and knockdown of LINC01089, the expression of PTEN in NSCLC cells was detected by Western blot

### LINC01089 affected the progression of NSCLC via targeting miR-152-3p

Next, we co-transfected miR-152-3p mimics into H1299 cells with over-expressed LINC01089, and the expressions of LINC01089, miR-152-3p and PTEN in H1299 cells were detected by qRT-PCR, and it was suggested that the expression of PTEN was induced by LINC01089, but partially reversed by the co-transfection of miR-152-3p (Fig. 6a-c). We further examined the proliferation, migration and invasion of H1299 cells. CCK-8, scratch healing and Transwell assays showed that after co-transfection of miR-152-3p mimics, the proliferation, migration and invasion of H1299 cells inhibited by LINC01089 were remarkably rescued (Fig. 6d-f). In addition, Western blot results indicated that overexpression of miR-152-3p attenuated the effects of LINC01089 overexpression on PTEN expression; on the other hand, down-regulation of miR-152-3p reversed the effects of LINC01089 knockdown on PTEN expression (Fig. 6g). These results exhibited that miR-152-3p could reverse the inhibitory effect of LINC01089 on malignant phenotype of NSCLC cells.

**Fig. 6:** LINC01089 affected the proliferation, migration and invasion of H1299 cells via miR-152-3p/PTEN axis. **a**-**c**: After miR-152-3p mimics were transfected into H1299 cells overexpressing LINC01089, the expressions of LINC01089, miR-152-3p and PTEN mRNA were detected by qRT-PCR. NS *P* > 0.05, *P < 0.05, **P < 0.01, ***P < 0.001. **d** CCK-8 assay was used to detect the proliferation of H1299 cells after transfection of miR-152-3p mimics into H1299 cells overexpressing LINC01089, *P < 0.05, **P < 0.01(vs. Vector); ^&^*P* < 0.05, ^&&^*P* < 0.01(vs. LINC01089/NC). **e** The migration ability of H1299 cells was measured by scratch assay after transfection of miR-152-3p mimics into H1299 cells overexpressing LINC01089, **P < 0.01. **f** After miR-152-3p mimics were transfected into H1299 cells overexpressing LINC01089, the invasive ability of H1299 cells was detected by Transwell assay. **P < 0.01. **g** Western blot was used to detect the regulatory effects of LINC01089 and miR-152-3p on the expression of PTEN in NSCLC cell lines

## Discussion

Cancer has become one of the major public problems that seriously threaten the health of people on a global scale. Although great progresses have been made in clinical treatments such as surgery, chemotherapy, radiotherapy and targeted therapy, NSCLC remains the leading cause of cancer-related deaths worldwide. Distal metastasis and recurrence were the major hurdles to improve the prognosis of patients [22]. Therefore, studying the mechanism of NSCLC progression is of great significance.

Recent studies have demonstrated that lncRNAs are involved in regulating the proliferation and metastasis of NSCLC cells. For example, lncRNA PDIA3P promotes proliferation and metastasis of NSCLC cells by modulating the Wnt/β-catenin signaling pathway [23]. In addition, lncRNA LBX2-AS1 promotes proliferation and metastasis of NSCLC cells via regulating Notch signaling, and its high expression suggests poor prognosis [24]. In this work, the expression of LINC01089 in NSCLC was investigated, and it was proved to be down-regulated in NSCLC tissues and cells, and its under-expression indicated unfavorable prognosis of the patients. We also probed the effects of LINC01089 on proliferation, migration and invasion of NSCLC cells with gain-of-function models and loss-of-function models. We found that LINC01089 overexpression could impede the proliferation, migration and invasion of NSCLC cells, while the knockdown of LINC01089 had the opposite effects. These results suggested that LINC01089 was a tumor suppressor in NSCLC, and its tumor-suppressive function found in our work is consistent with the previous report [13].

Accumulating studies have indicated that lncRNA can modulate the progression of NSCLC via sponging miRNA. For example, lncRNA CASC15 is up-regulated in NSCLC tissues and can facilitate the progression of NSCLC via targeting miR-130b-3p [25]. LncRNA FENDRR inhibits the progression of NSCLC by modulating the miR-761/TIMP2 axis [26]. In different cancers, the role of miR-152-3p is distinct. In glioma, prostate cancer, hepatocellular carcinoma, it exhibits antineoplastic activity[16, 17, 27]; while in chronic myeloid leukemia, it is oncogenic [28]. In lung cancer, the role of miR-152-3p is rarely studied in previous studies. It is reported that the low level of plasma miR-152-3p indicates poor prognosis of patients with squamous cell carcinoma [29]. However, its biological function remains unclear in NSCLC. A study has depicted that LINC00174 can function as the ceRNA of miR-152-3p to up-regulate SLC2A1 to promote the progression of glioma, which implying the crucial role of lncRNA in regulating the expression of miR-152-3p [30]. In this work, we demonstrated that miR-152-3p was up-regulated in NSCLC tissues, and LINC01089 could adsorb miR-152-3p to negatively regulate its expression. Moreover, we demonstrated that miR-152-3p could reverse the effects of LINC01089 on the biological behaviors of NSCLC cells. For the first time, our results indicated that miR-152-3p was an oncogenic miRNA in NSCLC.

MiRNAs promotes mRNA degradation or inhibits translation process to affect the progression of NSCLC by complementary pairing with the 3’UTR of the target mRNA. For example, miR-608 impedes proliferation and metastasis of NSCLC cells via targeting the BRD4 [31]. MiR-7-5p functions as a tumor suppressor o block the progression of NSCLC via targeting PAK2 [32]. The interaction between miR-152-3p and PTEN has been reported previously. In hepatocytes, down-regulated miR-152-3p disrupts hepatic glycogenesis by targeting PTEN [33]; tanshinone IIA inhibits apoptosis of cardiomyocytes by inducing miR-152-3p and thereby down-regulating PTEN [34]. In this study, we demonstrated that, PTEN, the famous tumor suppressor, was a target gene of miR-152-3p and negatively regulated by it in NSCLC, which was consistent with the previous reports [33, 34]. Additionally, we found that PTEN in NSCLC cells was positively regulated by LINC01089. Collectively, our results indicated that LINC01089 could inhibit the progression of NSCLC through regulating miR-152-3p/PTEN axis.

The current research has some limitations. Firstly, *in vivo* studies are important to further validate the function of LINC01089/miR-152-3p/PTEN axis in NSCLC progression. Additionally, whether LINC01089 can regulate other phenotypes of NSCLC cells (such as chemosensitivity and radiosensitivity) awaits further investigation. In breast cancer, LINC01089 functions as a tumor suppressor via regulating cell cycle regulators and wnt/β-catenin signaling [13]. A recent study also suggests that LINC01089 inhibits tumorigenesis and epithelial-mesenchymal transition of NSCLC via the miR-27a/SFRP1/Wnt/β-catenin axis [21]. These studies suggest that LINC01089 is a crucial regulator in Wnt/β-catenin signaling. It is also interesting to explore whether LINC01089 can regulate the progression of NSCLC via this mechanism or other mechanisms.

Taken together, our study confirms that LINC01089 can function as a tumor suppressor and impede the proliferation, migration and invasion of NSCLC cells through the miR-152-3p/PTEN axis. This work presents potential biomarkers and therapy targets for NSCLC, and help clarify the mechanism of NSCLC tumorigenesis and progression.

## Data Availability

The data used to support the findings of this study are available from the corresponding author upon request.
